RETRACTED

# Efficacy and Safety of Different Thermal Ablation Modalities for Papillary Thyroid Microcarcinoma: A Network Meta-Analysis

**DOI:** 10.1155/2022/9448349

**Published:** 2022-07-31

**Authors:** Lieming Wu, Xi Chen

**Affiliations:** ^1^Department of Thyroid and Breast Surgery, The PLA Navy Anqing Hospital, Anqing 246000, Anhui, China; ^2^Department of Thyroid and Breast Surgery, Anqing Municipal Hospital, Anhui, Anqing 246000, Anhui, China

## Abstract

**Background:**

Small thyroid-like carcinoma (PTMC) is one of the most common subtypes of thyroid cancer. The main treatment options include surgery and radiofrequency ablation (RFA), microwave ablation (MWA), and laser ablation (LA). Thermal ablation has the advantage of being less invasive and has fewer complications than traditional surgical treatment.

**Objective:**

The objective is to explore the efficacy and safety of PTMC by different thermal ablation modalities through a network meta-analysis.

**Methods:**

From the database establishment to October 2021, a computerized search of the Chinese Knowledge Infrastructure (CKNI), VIP Chinese Science and Technology Journal Full-Text Database (VP-CSJFD), WanFang Data journal article resource (WangFang), PubMed, the Cochrane Library, and Embase were performed to include the different methods of thermal ablation for small thyroid carcinoma. A retrospective study of different methods of thermal ablation of small thyroid carcinoma was included.

**Results:**

A total of 12 retrospective studies involving 1,926 patients with PTMC were included, all of which were of high quality. This study mainly involved RFA, MWA, LA, and ethanol combined with radiofrequency ablation (EA + RFA). Network meta-analysis showed no significant difference between interventions (*p* > 0.05) in terms of recurrence rate.

**Conclusions:**

Surgical resection may be the measure with the lowest recurrence rate after treatment of PTMC, LA may be the measure with the lowest incidence of complications after treatment, and RFA may be the measure with the least length of hospital stay, operation time, and postoperative lymph node metastasis rate. However, due to the limitations of network meta-analysis, this result still needs to be treated with caution, and more high-quality, large-sample clinical studies are recommended for further verification.

## 1. Introduction

In recent years, with improved diagnostic techniques, there has been a global increase in the incidence of PTMC, a thyroid-like microcarcinoma (PTMC) of less than 10 mm in diameter, which is less aggressive and has a good prognosis [1, 2]. Although studies [3, 4] have shown recurrence and metastasis rates of 20% to 50% in patients with PTMC, in specific guidelines developed by the American Association of Thyroid Physicians in 2015 for the surgical approach to differentiated thyroid carcinoma, PTMC is considered to be of low-risk and patients may opt for follow-up observation and dynamic evaluation without immediate surgery [5]. Due to increased patient health awareness, most patients have a higher psychological burden after diagnosis and choose to use medical treatment for early intervention. Surgery remains the main treatment for PTMC [6]. The traditional surgical treatment produces surgical scars, the possibility of intraoperative laryngeal return nerve, parathyroid damage, and lifelong postoperative levothyroxine administration, which are often not easily accepted by patients.

RETRACTED

In addition to surgical excision of the lesion, nonsurgical treatment modalities are already available for PTMC. Thermal ablation is a surgical procedure that uses heat to induce focal tissue coagulation and necrosis. Initially used only for benign tumors, it is now recognized for the treatment of a wide range of diseases [7–9]. PTMC patients are gradually participating in thermal ablation with good results [10]. Commonly used thermal ablations include radiofrequency ablation (RFA), microwave ablation (MWA), and laser ablation (LA). Many studies [11–13] have reported the effectiveness and safety of different thermal ablation methods for the treatment of PTMC. Therefore, this paper uses network meta-analysis to evaluate the efficacy of various therapeutic measures such as RFA, LA, and MWA, and select the thermal ablation method with the best therapeutic effect to provide theoretical guidance for the clinical selection of therapeutic measures for small thyroid carcinoma.

## 2. Materials and Methods

### 2.1. Literature Search Strategy

Two investigators searched independently according to the search rules of each database.

#### 2.1.1. Search the Database

The databases of China National Knowledge Infrastructure (CKNI), VIP Chinese Science and Technology Journal Full-text Database (VP-CSJFD), Wanfang Database (WangFang), PubMed, the Cochrane Library, and Embase were searched by computer.

#### 2.1.2. Search Terms

The search terms are “Thermal ablation,” “Laser ablation,” “Radiofrequency ablation,” “Microwave ablation,” and “Thyroid papillary carcinoma.”

#### 2.1.3. Search Time

Each database was built until October 2021.

#### 2.1.4. Literature Search Strategy

The search method is subject terms combined with free terms, with PubMed: ((“Thyroid Cancer, Papillary”(Mesh)) OR (Papillary Thyroid Cancer (Title/Abstract)) OR (Papillary Carcinoma Of Thyroid (Title/Abstract)) OR (Papillary Thyroid Carcinoma (Title/Abstract)) OR (Familial Nonmedullary Thyroid Cancer (Title/Abstract)) OR (Nonmedullary Thyroid Carcinoma (Title/Abstract)) OR (Papillary thyroid microcarcinoma (Title/Abstract)) OR (Thyroid micropapillary carcinoma (Title/Abstract))) AND ((“Radiofrequency Ablation”(Mesh)) OR (Radio-Frequency Ablation (Title/Abstract)) OR (Radio Frequency Ablation (Title/Abstract)) OR (Thermal ablation (Title/Abstract)) OR (Laser ablation (Title/Abstract)) OR (Microwave ablation (Title/Abstract))).

RETRACTED

### 2.2. Inclusion and Exclusion Criteria

#### 2.2.1. Inclusion Criteria

1. The study type was a cohort study of thermal ablation treatment of microscopic thyroid carcinoma;
2. The observation group intervened with one or more of the three thermal ablation treatments, and the control group was surgical resection, ethanol ablation, or other thermal ablation treatments different from the observation group;
3. The diagnosis of thyroid carcinoma was confirmed by pathology, and microscopic carcinoma was defined as ≤10 mm in diameter;
4. The study outcome indicators included recurrence rate, lymph node metastasis rate, complication rate, length of hospital stay, and duration of surgery.

#### 2.2.2. Exclusion Criteria

1. Repeated publication, no original text found in the literature;
2. Review category, experience summary, case report, meeting, meta-analysis, etc.;
3. Disease diagnosis inconsistent with papillary thyroid microcarcinoma;
4. Interventions do not include thermal ablation.

### 2.3. Literature Screening and Data Extraction

(1) The retrieved literature was imported into EndNote software, the repeated literature was deleted after checking, and then two investigators deleted the unqualified literature by reading the titles and abstracts of the remaining literature according to the above proposed inclusion and exclusion criteria; (2) For the remaining literature, two investigators read the full text in detail and deleted the literature, not including outcome measures, incomplete data or repeated data result; (3) To ensure the accuracy of data and the rigor of the study, two investigators extracted the relevant data, and the extracted contents mainly included: the study authors, publication year, baseline conditions, intervention measures, and outcome measures, which were integrated and checked with each other after the data were extracted and perfected. In case of any disagreement during the above process, third-party experts with many years of experience in evidence-based medicine shall be invited for joint judgment. The judgment results of the third-party experts shall be taken as the final results.

### 2.4. Literature Quality Evaluation Method

Newcastle-Ottawa Scale (NOS) was used for quality evaluation of the included literature. The scale consists of three aspects of assessment: the selection method of the case-control group, the comparability of the case-control group, and the assessment method of contact exposure. The total score of each piece of literature is 9 points, (5–9) points for high-quality literature and less than 5 points for low-quality literature.

RETRACTED

### 2.5. Statistical Methods

Network meta-analysis was performed using Stata 16.0 software. The thicker the line in the relationship of evidence plot of included studies, the greater the number of included studies. The overall agreement between direct and indirect evidence was analyzed using an inconsistency test, and *p* > 0.05 was considered to indicate inconsistency, fitting the agreement model and vice versa. Local inconsistency tests were performed using nodal splitting for direct and indirect comparisons, with *p* < 0.05 indicating local inconsistency.

## 3. Results

### 3.1. Literature Results

After a systematic search, 1,469 pieces of literature were obtained, 925 pieces were obtained after EndNote X9 software was reweighted, and 60 pieces of literature were obtained after excluding irrelevant literature. In uncontrolled experimental studies, 27 pieces of literature were obtained after reading the titles and abstracts of the remaining literature. Then, 12 pieces of literature [14–25] with 1,926 patients were finally included after excluding the literature with missing outcome measures (*n* = 5), incomplete data reporting (*n* = 3), and low-quality literature (*n* = 7) after reading the full text (Figure 1).

### 3.2. Basic Characteristics and Quality Evaluation of the Included Literature

Of the 12 articles included in this study, six were in English and 6 in Chinese. This study mainly involves radiofrequency ablation (RFA), microwave ablation (MWA), laser ablation (LA), and ethanol combined with radiofrequency ablation (EA + RFA). All the study results are from the Chinese region, retrospective cohort studies. The basic characteristics were comparable among the studies regarding age, gender, and diameter of PTMC of the patients included in the study. The NOS scores of all 12 articles were ≧ 5, indicating that the quality of the included articles was high (Table 1).

### 3.3. Network Meta-analysis Results

#### 3.3.1. Evidence Network

The network evidence diagram (Figure 2(a)) of recurrence rate, complication rate, lymph node metastasis rate, length of hospital stay, and operation time after PTMC treatment with three thermal ablation methods shows that: there is a direct or indirect comparison between different interventions, which has the basic condition for network meta-analysis.

RETRACTED

#### 3.3.2. Consistency Test

The results showed no inconsistency (*p* > 0.05) between direct and indirect comparisons in terms of recurrence rate, the complication rate of lymph node metastasis, length of hospital stay, and operative time, with good local agreement. Therefore, consistency model analysis could be used.

#### 3.3.3. Network Meta-Analysis

*(1) Recurrence Rate*. Ten pieces of literature [14, 15, 17–23, 25] reported the recurrence rate after thermal ablation for PTMC. The interventions included LA, MWA, RFA, and surgery. The results of the reticular meta-analysis showed: comparison between any two interventions had no statistical significance (*p* > 0.05). SUCRA results showed: surgery (62.1%) > LA (51.4%) > MWA (51.0%) > RFA (35.6%), suggesting that surgery may be the intervention with the lowest recurrence rate after treatment of PTMC, followed by LA (Table 2 and Figure 3(a)).

*(2) Lymph Node Metastasis Rate*. Nine pieces of literature [14, 15, 17–21, 23, 25] reported lymph node metastasis rate after thermal ablation for PTMC. Intervention measures included LA, MWA, RFA, and surgery. Reticular meta-analysis results showed: comparison between any two interventions had no statistical significance (*p* > 0.05). SUCRA results showed: RFA (68.7%) > LA (59.6%) > MWA (37.3%) > surgery (34.5%), suggesting that RFA may be the intervention with the lowest rate of lymph node metastasis after treatment of PTMC, followed by LA (Table 3 and Figure 3(b)).

*(3) Complication Rate*. Twelve pieces of literature [14–25] reported the incidence rate of complications after thermal ablation for PTMC. The intervention measures included EA-RFA, LA, MWA, RFA, and surgery. The reticular meta-analysis results showed: the incidence rate of complications after EA-RFA, LA, MWA, and RFA was lower than those after surgery (*p* < 0.05). The other pairwise comparisons had no statistical significance (*p* > 0.05). SUCRA results showed: LA (86.0%) > EA + RFA (66.1%) > MWA (42.2%) > RFA (42.2) > surgery (0.4%), suggesting that LA may be the intervention with the lowest complication rate after treatment of PTMC, followed by EA + RFA (Table 4 and Figure 3(c)).

*(4) Length of Stay*. Six pieces of literature [17–20, 22, 25] reported the length of stay after thermal ablation for PTMC. The intervention measures included LA, MWA, RFA, and surgery. The reticular meta-analysis results showed: the length of hospital stays after LA, MWA, and RFA were all significantly longer than those after surgery (*p* < 0.05), and the other pairwise comparisons had no statistical significance (*p* > 0.05). The results of SUCRA showed: RFA (82.7%) > MWA (60.0%) > LA (56.6%) > Surgery (0.1%), suggesting that RFA may be an intervention for the shortest length of stay after the treatment of PTMC, followed by MWA (Table 5 and Figure 3(d)).

*(5) Operation Time*. Seven pieces of literature [17–22, 25] reported the operation time of thermal ablation for PTMC. The intervention measures included LA, MWA, RFA, and surgery. The network meta-analysis results showed that: the length of hospital stays after LA, MWA, and RFA were significantly longer than those after surgery (*p* < 0.05). The results of SUCRA showed: RFA (86.2%) > MWA (58.4%) > LA (55.0%) > surgery (0.4%), suggesting that RFA may be an intervention for the shortest operation time after the treatment of PTMC, followed by MWA (Table 6 and Figure 3(e)).

RETRACTED

### 3.4. Publication Bias

It can be found from the funnel plot of recurrence rate, lymph node metastasis rate, complication rate, length of hospital stay, and operation time that each point is scattered and asymmetrically incomplete, suggesting that there may be some publication bias. There is a scattered point distribution at the bottom of the funnel plot of each study indicator, indicating that there is a small sample effect (Figure 4(a)).

## 4. Discussion

The American Thyroid Association [26] supports active surveillance of patients with low-risk PTMC, especially those with high surgical risk or short life expectancy. Papillary and follicular carcinomas are differentiated thyroid carcinomas derived from the follicular epithelium and account for 90% of thyroid cancers [27]. Papillary carcinoma has a good prognosis, with a 20-year mortality rate of 1% to 2% [28]. Therefore, most diagnosed patients still tend to eliminate cancer. In addition to active surveillance, surgery is the most common traditional treatment, while thermal ablation is an emerging minimally invasive method.

There are no official associations and guidelines internationally recommending thermal ablation as the first-line treatment for PTMC. Several clinical studies of thermal ablation for primary PTMC have also been published internationally, the vast majority of which are from China. In these studies, the main inclusion criteria for thermal ablation of PTMC included: (1) PTC confirmed by puncture pathology and a single lesion no larger than 10 mm. (2) No peripheral tissue or extraglandular invasion of the nodule and no neck or distant metastasis of the lymph nodes. (3) The patient is objectively unable to undergo surgery or subjectively refuses surgery.

The therapeutic value of RFA for benign thyroid nodules has been generally recognized. However, whether RFA can treat PTMC is still controversial. Some scholars believe that for low-risk PTMC patients, RFA can be used as an alternative to surgical treatment. Kim et al. [29, 30] evaluated the effect of RFA in 74 patients with 84 lesions of PTMC, of which 13 underwent a second treatment, with a complication rate of 1.4%, complete tumor disappearance at two and five years after surgery of 98.8% and 100%, and no local tumor progression, lymph node metastasis or distant metastasis during the follow-up period. Kim et al. [31] and Jeong et al. [32] in Asan Hospital, Korea, performed radiofrequency ablation on 6 cases of PTMC each and found that the lesion volume became significantly smaller after an average observation of 48.5 and 19.3 months, respectively, without any metastasis or recurrence. MWA was also effective in treating benign thyroid nodules, significantly reducing the operation time and length of hospital stay [33].

RETRACTED

Compared with Surgery, MWA was associated with fewer mean hospital stays, costs, mean blood loss, and surgical incision healing time [34]. Three domestic studies have explored the application of microwave ablation in the treatment of PTMC. Microwave ablation was performed on more than 290 PTMC cancer foci in 21 cases, 15 cases, 46 cases, and 185 patients, respectively. The observation ranged from 11 to 42 months. No tumor recurrence or residual was found [35–37]. Compared with laser ablation, radiofrequency and microwave ablation are characterized by “mobile ablation,” which is more flexible and easier to operate. In 2011, Papini et al. in Italy first applied the laser to the treatment of PTMC patients and confirmed the safety and efficacy of LA treatment. Papini et al. performed ultrasound-guided laser ablation in an 81-year-old PTMC patient with decompensated cirrhosis, renal failure, and after breast cancer radiation therapy. The nodule changed from the initial 8 mm to 4 mm after 24 months, and no cancer cells were observed after another fine-needle aspiration cytology [38]. Two years later, Valcavi et al. [39] in Italy, after fully informed communication, performed laser ablation after general anesthesia in three patients diagnosed with PTMC and immediately underwent total thyroidectomy. Postoperative pathology confirmed that the tumor tissue had been destroyed and carbonized with complete disappearance of activity but one of the patients had one lymph node metastasis. Since then, Chinese scholars have carried out clinical studies on a large number of cases. Zhou et al. [40] retrospectively analyzed the effect of ultrasound-guided laser ablation in 30 patients with PTMC diagnosed by fine-needle aspiration cytology, in which 29 patients completed the treatment in a single time under local anesthesia, and the other patient underwent contrast-enhanced ultrasound for the second ablation after laser ablation. After a follow-up of 24 months, it was found that the ablation lesions disappeared in 10 patients, 20 patients still had scar-like lesions, and no regrowth, recurrence, or distant metastasis of the ablated lesions was found.

RETRACTED

There have been no studies directly comparing the efficacy and safety of these three techniques, laser, radiofrequency, and microwave ablation, for the treatment of PTMC. This study compared the efficacy and safety of RFA, MWA, and LA in terms of recurrence rate, lymph node metastasis rate, complication rate, operation time, and length of hospital stay after thermal ablation for PTMC. We found that surgical resection may be the measure with the lowest recurrence rate after treatment of PTMC, LA may be the measure with the lowest incidence of complications after treatment, and RFA may be the measure with the least length of hospital stay, operation time, and postoperative lymph node metastasis rate. The incidence of complications, operation time, and hospital stay after RFA, MWA, and LA were significantly lower than those after surgery, and the differences had statistical significance (*p* < 0.05). First, there is still no optimal consensus on the indications of thermal ablation therapy for PTMC. Second, the necessity and feasibility of distinguishing the risk of PTMC progression before ablation are still worth thinking about. The active observation studies of PTMC by Korean and Japanese research teams have shown that age of less than 40 years, and higher initial serum thyroid-stimulating hormone levels are important risk factors for PTMC progression in active observation [41, 42].

Furthermore, the important role of thermal ablation in the treatment of PTMC is the absence of cervical lymph node metastasis. In the face of so many lymph node metastases, the sensitivity of ultrasound in the diagnosis of abnormal lymph nodes in the central and lateral cervical regions is 25% to 60% and 70% to 95%, and the diagnostic sensitivity can be improved by 15% after combined cervical CT [43].

Our study is the first to investigate the differences among the three thermal ablation treatment modalities using network meta-analysis but this study also has some limitations. Our conclusions are mainly derived from indirect evidence, and the strength of evidence of the findings is weaker than that derived from direct evidence. In addition, the original literature included in this study was a retrospective cohort study. The quality of original literature was not as good as that of randomized controlled trials to a certain extent, which also affected the reliability of the results [44].

RETRACTED

## 5. Conclusion

Combined with the available clinical reports and studies, thermal ablation has shown efficacy and safety in the treatment of low-risk PTMC and is expected to be a new option for the first-line treatment of some low-risk PTMC patients. Due to limited research data, evaluation of the advantages and disadvantages of the three thermal ablation techniques still requires further validation in large-sample, multicenter, prospective randomized controlled trials.

## Figures and Tables

**Figure 1:** The literature screening flow chart.

**Figure 2:** (a) Network evidence graph for recurrence rate. (b) Network evidence plot for lymph node metastasis rate. (c) Network evidence plot for complication rate. (d) Network evidence plot for length of stay. (e) Network evidence plot for surgical time.

**Figure 3:** (a) Probability plot of recurrence rate ordered. (b) Probability ranking plot for lymph node metastasis rate. (c) Probability ranking plot of complication rate. (d) Probability plot for length of stay. (e) Probability plot for procedure time.

**Figure 4:** (a) Funnel plot of recurrence rate. (b) Funnel plot of lymph node metastasis rate. (c) Funnel plot of complication rate. (d) Funnel plot of the length of hospital stay. (e) Funnel plot of operation time.

**Table 1:** The basic characteristics and quality evaluation of literature.

Author	Country	Year	Type of study	Sex(M/F)	Age(s)	Sample sizes	Interventions	PTMC diameters (mm)	Outcomes	NOS scores
Shen et al. [14]	China	2019	Cohort study	16/29	43.7 ± 6.6	45	RFA	6.12 ± 1.23	①②③	5
				24/28	40.5 ± 7.8	52	MWA	6.21 ± 1.16		

Sun and Dong [15]	China	2018	Cohort study	20/27	42.66 ± 4.19	47	RFA	6.17 ± 1.11	①②③	6
				18/21	43.09土5.14	39	MWA	6.04 ± 1.2		

Gong et al. [16]	China	2019	Cohort study	26/53	49.32 ± 7.48	75	MWA	6.31 ± 1.71	③	5
				23/52	49.67 ± 7.39	79	RFA	6.77 ± 1.68		
				20/53	48.86 ± 7.42	73	Surgery	6.28 ± 1.69		

Feng et al. [17]	China	2019	Cohort study	26/76	47.4 ± 11.2	102	RFA	5.9 ± 1.7	①②③④⑤	5
				23/92	43.9 ± 10.7	115	Surgery	6.3 ± 2.2		

Zhou et al. [18]	China	2020	Cohort study	14/36	42.16 ± 10.28	50	Surgery	4.30 ± 1.25	①②③④⑤	5
				11/40	44.72 ± 9.94	51	MWA	4.46 ± 1.39		

Yao et al. [19]	China	2020	Cohort study	19/101	45.86 ± 8.30	120	MWA	5.89 ± 1.12	①②③④⑤	5
				22/98	46.02 ± 8.11	120	Surgery	5.96 ± 1.05		

Li et al. [20]	China	2018	Cohort study	14/32	43.63 ± 9.27	46	MWA	4.49 ± 1.55	①②③④⑤	7
				13/33	49.59 ± 9.0	46	Surgery	4.29 ± 1.37		

Xiao et al. [21]	China	2021	Cohort study	19/72	40.7 ± 9.3	91	RFA	1.4 ± 0.2 cm	①②③⑤	5
				23/68	40.2 ± 10.4	91	Surgery	1.4 ± 0.2 cm		

Zhou et al. [22]	China	2020	Cohort study	7/26	37.9 ± 10.1	33	MWA	5.0 ± 1.4	①②③④⑤	6
				11/23	41.8 ± 13.4	34	LA	4.5 ± 1.6		

Li et al. [23]	China	2019	Cohort study	36/132	47.36 ± 10.75	168	MWA	4.67 ± 1.65	①②③	6
				29/114	49.18 ± 11.41	143	Surgery	4.59 ± 1.77		

Zhu et al. [24]	China	2020	Cohort study	16/28	45 ± 17	44	EA + RFA	5.78 ± 1.55	③	6
				15/29	46 ± 17	44	RFA	5.89 ± 1.37		

Song et al. [25]	China	2021	Cohort study	18/97	44.9 ± 10.4	115	RFA	6.5 ± 1.9	①②③④⑤	7
				19/84	45.4 ± 9.9	103	Surgery	6.9 ± 1.6		

① Recurrence Rate; ② Lymph Node Metastasis Rates; ③ Complication Rates; ④ Length of Stay; ⑤ Surgical Time.

RETRACTED

**Table 2:** The network meta-analysis of recurrence rate after different thermal ablation methods for PTMC [RR, 95% CI].

LA			
0.97 (0.02,47.53)	MWA		
0.77 (0.01,47.76)	0.79 (0.20,3.18)	RFA	
1.12 (0.02,60.71)	1.15 (0.46,2.86)	1.46 (0.43,4.97)	Surgery

**Table 3:** Network meta-analysis of lymph node metastasis rates after different thermal ablation modalities for PTMC [RR, 95% CI].

LA			
0.48 (0.01,35.56)	MWA		
0.97 (0.02,47.56)	2.03 (0.32,13.01)	RFA	
0.46 (0.01,32.10)	0.96 (0.18,5.08)	0.47 (0.09,2.61)	Surgery

**Table 4:** The network meta-analysis of complication rates after different thermal ablation modalities for PTMC [RR, 95% CI].

EA-RFA				
2.51 (0.18,34.67)	LA			
0.81 (0.22,2.93)	0.32 (0.03,3.20)	MWA		
0.67 (0.25,1.80)	0.27 (0.02,3.03)	0.82 (0.36,1.86)	RFA	
0.18 (0.05,0.61)	0.07 (0.01,0.78)	0.23 (0.13,0.40)	0.27 (0.14,0.55)	Surgery

**Table 5:** The network meta-analysis of the length of hospital stays after different thermal ablation modalities for PTMC [SMD, 95% CI].

LA			
0.19 (−1.95, 2.32)	MWA		
0.86 (−2.04, 3.76)	0.67 (−1.30, 2.64)	RFA	
−3.65 (−6.12, −1.18)	−3.84 (−5.09, −2.58)	−4.51 (−6.03, −2.99)	Surgery

**Table 6:** The network meta-analysis of procedure time after different thermal ablation modalities for PTMC [WMD, 95% CI].

LA			
3.56 (−33.08, 40.19)	MWA		
17.54 (−29.80, 64.89)	13.99 (−16.41, 44.39)	RFA	
−49.04 (−91.26, −6.82)	−52.59 (−74.05, −31.14)	−66.58 (−88.16, −45.01)	Surgery

## Data Availability

The experimental data used to support the findings of this study are available from the corresponding author upon request.
